The article "Rapid-Onset Antidepressant-Like Effect of Nelumbinis semen in Social Hierarchy Stress Model of Depression" was published in 2022. Journal: Evid Based Complement Alternat Med.

# Rapid-Onset Antidepressant-Like Effect of *Nelumbinis semen* in Social Hierarchy Stress Model of Depression

**DOI:** 10.1155/2022/6897359

**Published:** 2022-05-29

**Authors:** Jihwan Shin, Jeonghun Lee, Junhyuk Choi, Byung-Taek Ahn, Sang Chul Jang, Seung-Won You, Do-Yeon Koh, Sungho Maeng, Seung-Yun Cha

**Affiliations:** ^1^Graduate School of East-West Medical Science, Kyung Hee University, Yong-in 17104, Republic of Korea; ^2^AgeTech-Service Convergence Major, Graduated School of East-West Medical Science, Kyung Hee University, Young-in 17104, Republic of Korea

## Abstract

Depression is a disease with increasing prevalence worldwide, and it is necessary to develop a therapeutic agent with better efficacy than existing antidepressant drugs. Antidepressants that act on the glutamatergic nervous system, such as ketamine, have a rapid-onset antidepressant effect and are effective against treatment-resistant depression. However, because of the addictive potential of ketamine, alternative substances without psychological side effects are recommended. In particular, many natural compounds have been tested for their antidepressant effects. The antidepressant effects of *Nelumbinis semen* (NS) have been tested in many studies, along with the various actions of NS on the glutamatergic system. Thus, it was expected that NS might have a rapid-onset antidepressant effect. To test the antidepressant potential, despair and anhedonic behaviors were measured after administering NS to mice exposed to social hierarchy stress (SHS), and biochemical changes in the prefrontal cortex and hippocampus were analyzed. NS reduced despair-like responses in the forced swim test and tail suspension test. Mice exposed to SHS showed depression-like responses such as increased despair, reduced hedonia, and an anxiety-like response in the novelty suppressed feeding test. NS, but not fluoxetine, improved those depression-like behaviors after acute treatment, and NBQX, an AMPA receptor blocker, inhibited the antidepressant-like effects of NS. The antidepressant-like effect of NS was related to enhanced phosphorylation of mTOR in the prefrontal cortex and dephosphorylation of GluR1 S845 in the hippocampus. Since NS has shown antidepressant-like potential in a preclinical model, it may be considered as a candidate for the development of antidepressants in the future.

## 1. Introduction

Depression is one of the most prevalent health concerns, and unlike other diseases for which preventive treatment has been established, the number of patients is not expected to decrease soon [1]. This is because depression is caused by a combination of many physical, mental, and social factors [2]. Various methods were developed to treat depression; however, none of these methods could completely cure depression. Especially, conventional antidepressants are only effective in some patients, and clinical studies (STAR^*∗*^D) have pointed out that they offer limited efficacy and a low rate of full remission [3, 4].

The article "Rapid-Onset Antidepressant-Like Effect of Nelumbinis semen in Social Hierarchy Stress Model of Depression" was published in 2022. Journal: Evid Based Complement Alternat Med.

Interest in antidepressants that act on the glutamatergic system has been increasing since the discovery that a subanesthetic dose of ketamine has a rapid and lasting antidepressant effect [5, 6]. The antidepressant effect of ketamine and substances acting on the glutamatergic system was related in NMDA-to-AMPA throughput, mTOR activation, and inhibition of the reward stimulation circuit by the lateral habenula [7–9]. In addition, these drugs are effective in treatment-resistant depression, for which existing antidepressants do not work, so they are expected to replace existing antidepressants in the future [10].

*Nelumbo nucifera* Gaertner (NNG), a perennial aquatic herb, is common in Korea, Australia, China, India, Iran, Japan, and regions of southeast Asia [11]. Almost all parts of NNG, i.e., leaves, flowers, seeds, roots, rhizomes, and embryo, are used as food garnishes and for various medicinal purposes. The seed of NNG, *Nelumbinis semen* (NS), was traditionally used as a sedative, antipyretic, and hemostatic to treat disorders such as insomnia, fevers, hypertension, arrhythmia, and postmenopausal depression [12–14]. It is also consumed as health-promoting foods that can treat ailments such as skin diseases and tissue inflammation and act as a poison antidote, astringent, emollient, and diuretic [15,16]. NS contains alkyl 4-hydroxybenzoates, bisbenzylisoquinoline alkaloids, benzylisoquinoline alkaloids, aporphine, and proaporphine alkaloids [17–21]. In previous studies, NS was shown to have antidepressant-like effects in rats; those effects were associated with local cholinergic and dopaminergic or noradrenergic neurotransmission in the hippocampus and prefrontal cortex [22, 23].

A recent publication has demonstrated that preparations containing NS have antidepressant effects via activation of the brain-derived neurotrophic factor through the Rac1-cofilin signaling pathway [24]. The stem part of NS exhibited antidepressant activity through NCAM and GAP-43 regulation [25]. Like the NMDA receptor antagonist ketamine, glutamatergic system changes are among the known effects of NS. It protected against glutamate-induced apoptosis in HT22 cells [26]. The learning and memory improvement effects of NS were associated with mTOR-induced neurogenesis enhancement in the hippocampal dentate gyrus [27]. Also, neferine, a component of NS, reduces hypoxic damage by activating the Akt/mTOR pathway [28]. On the other hand, in lung cancer cell lines, NS inhibited the PI3K/AkT/mTOR pathway [29]. As such, NS was expected to have a rapid antidepressant effect by being involved in the glutamatergic system and the mTOR pathway. Since NS exhibits different effects in each tissue, it is necessary to study whether NS would show a rapid-onset antidepressant effect.

The article "Rapid-Onset Antidepressant-Like Effect of Nelumbinis semen in Social Hierarchy Stress Model of Depression" was published in 2022. Journal: Evid Based Complement Alternat Med.

Animal models to test the efficacy of antidepressant drugs are based on testing the construct validity of depressive symptoms such as behavioral despair and anhedonia and then determining whether the test drug improves those symptoms [30]. Among the depression models, rapid-onset antidepressant effects can be tested in models that do not respond to short-term but only to long-term administration of conventional antidepressants. In other words, if short-term administration of a drug improves depressive symptoms in those models, it can be said to have rapid antidepressant effects [8]. Appropriate depression models for those tests include learned helplessness, early life stress, social defeat stress, chronic unpredictable stress, and olfactory bulbectomy [31]. Also, in the novelty suppressed feeding test (NSFT), a decrease in feeding latency upon short-term administration of a test drug is considered to have an anti-anxiety effect, whereas a decrease in latency upon long-term administration is considered to have an antidepressant effect [32].

The model used in this study, the social hierarchy stress (SHS) model, forcibly puts animals that have a high rank in the social hierarchy into a low-rank state [33]. Subordinate males living in social hierarchies had significantly higher levels of plasma corticosterone than alpha males and pair-housed subordinate males [34]. Lowering an animal from a high rank to a low rank is a strong stressor that can induce depressive symptoms [35]. Rats maintaining a stable dominant status are more susceptible to the impact of status loss and showed more depressive behaviors, which were normalized by taking antidepressants for 3 weeks [36]. In addition, the socially dominant mouse is more vulnerable to chronic social defeat stress (CSDS) exposure than the subordinate mouse [37, 38]. The advantage of SHS as a depression model is that it requires less contact during the modeling process, and no direct physical harm is required, unlike the CSDS model [39].

Therefore, in this study, the SHS mice model was used to evaluate the antidepressant-like efficacy of NS on behavioral despair, anhedonia, and NSFT latency in comparison with the conventional antidepressant. We also measured whether the antidepressant effect of NS was inhibited by an AMPA receptor antagonist and measured the phosphorylation of mTOR and GluR1 in the prefrontal cortex and hippocampus.

The article "Rapid-Onset Antidepressant-Like Effect of Nelumbinis semen in Social Hierarchy Stress Model of Depression" was published in 2022. Journal: Evid Based Complement Alternat Med.

## 2. Materials and Methods

### 2.1. Animals and Experimental Groups

Eight-week-old male C57Bl/6 mice were purchased from Daehan Bio-link (Chungbuk, Korea) (*n* = 24 for cohort 1, *n* = 52 for cohort 2, and *n* = 24 for cohort 3). The animals were housed 4 to 6 per cage in climate-controlled quarters (24 ± 1°C, 55 ± 5% relative humidity) maintained with a 12 h light : 12 h dark cycle. The animals were provided with standard rodent chow and water ad libitum. After a week of habituation, the mice were randomly divided into experimental groups. The mice in cohort 1 were assigned to the following groups: vehicle (*n* = 6): DW p.o.; 0.1 mg/kg (*n* = 6): NS 0.1 mg/kg p.o.; 1 mg/kg (*n* = 6): NS 1 mg/kg p.o.; and 10 mg/kg (*n* = 6): NS 10 mg/kg p.o. The mice in cohort 2 were assigned to the following groups: normal (*n* = 4): not exposed to SHS + DW p.o.; vehicle (*n* = 4): exposed to SHS + DW p.o.; NS (*n* = 4): exposed to SHS + NS 1 mg/kg p.o.; and fluoxetine (*n* = 4): exposed to SHS + fluoxetine 10 mg/kg i.p. The mice in cohort 3 were assigned to the following groups: vehicle (*n* = 6): DW p.o.; NS (*n* = 6): NS 1 mg/kg p.o.; NBQX (*n* = 6): NBQX 10 mg/kg i.p.; and NS + NBQX (*n* = 6): NS 1 mg/kg p.o. and NBQX 10 mg/kg i.p. The experimental procedures are schematically outlined in Figure 1. All animal studies were conducted in accordance with the NIH Guide for the Care and Use of Laboratory Animals. The protocols were approved by the Institutional Animal Care and Use Committee of Kyung Hee University (KHUASP(GC)-19-040).

### 2.2. Preparation of NS Extract

Dried NS was purchased from Nong Lim Saengyak (Seoul, Korea). The NS (1.5 kg) were boiled at 121°C for 4 hours in eight times as much distilled water than NS by weight to produce an extract. After filtering the extract, the filtrate was decompressed to vapor in a rotary evaporator and freeze-dried. The yield of the extract was 36.7% (w/w).

### 2.3. Drug Administration and Treatment

The mice received a single oral administration of vehicle (DW) or NS extract (0.1, 1, and 10 mg/kg) dissolved in DW. Fluoxetine (10 mg/kg, Mallinckrdt Inc., St. Louis, MO, USA) was injected intraperitoneally 30 minutes before the test. NBQX (10 mg/kg, i.p., Tocris Bioscience, Bristol, UK) was given 30 minutes before administration of the NS extract.

### 2.4. Creating Model Animals (Social Hierarchy Stress Model)

This model is based on the dominance hierarchy. It induces SHS by using social defeat; that is, the dominance of a higher status individual is destroyed by a lower status individual [33]. This experiment used transparent acrylic tubes (30 cm long, 3.0 cm outer diameter, and 2.4 cm inner diameter). On the first day, short transparent acrylic tubes (10 cm long, 3.0 cm outer diameter, and 2.4 cm inner diameter) were placed in the home cages of each group. On the second and third days, the experimental long transparent acrylic tubes were placed in the cages to allow the mice to become accustomed to passing through the tube at both ends. After that, the dominance hierarchy in each group of four mice was determined by allowing pairs of them to enter the tube from each end. In each pair, the one that backed out of the tube first was considered to be lower in the social hierarchy than the one that walked out forward. If dominance was not determined within 2 minutes, those mice were excluded from the test. The mouse that won the test four times in a row was considered to have the highest status. To induce SHS, the highest status mouse was put in the tube from one end while a lower status mouse was placed on the other end, and then both ends were closed. In this situation, the lower rank mouse, finding it impossible to escape, might instead attack the higher rank mouse. The defeated dominant mice were the SHS model animals used for the cohort 2 experiments. A sucrose preference test was conducted to see whether the social stress model was created, and then behavioral tests were implemented, as shown in Figure 1 (Cohort 2).

The article "Rapid-Onset Antidepressant-Like Effect of Nelumbinis semen in Social Hierarchy Stress Model of Depression" was published in 2022. Journal: Evid Based Complement Alternat Med.

### 2.5. Behavioral Tests

#### 2.5.1. Novelty Suppressed Feeding Test

The mice were fasted for 24 hours before the experiment started. For this test, a single food pellet was placed at the corner (60 cm × 60 cm) of a dimly lit (<20 lux) Plexiglas test chamber. The latency to feeding was measured for 5 minutes. If the mice had not eaten the food within 5 minutes, the feeding latency was considered to be 5 minutes. In this test, nonfeeding behaviors (e.g., touching and smelling) were not considered as eating.

#### 2.5.2. Tail Suspension Test (TST)

Each mouse was suspended 45 cm above the floor by adhesive tape placed approximately 1 cm from the tip of the tail. The movement of the mice was filmed for 6 minutes, and immobility was measured through a review of the video footage by a researcher blinded to the research condition. Immobility was defined as the absence of any limb or body movement with the exception being if mice climbed their own tails.

#### 2.5.3. Forced Swimming Test (FST)

A Plexiglas cylinder (35 cm high and 20 cm in diameter) was filled with water to a height of 20 cm (±22°C) and the movement of mice was filmed for 6 minutes. During the 6-minute test session, immobility during the 4 minutes, from minutes two to six, was measured by a researcher blinded to the research condition. Immobility was defined as the minimal movement required for a mouse to keep its head above water.

The article "Rapid-Onset Antidepressant-Like Effect of Nelumbinis semen in Social Hierarchy Stress Model of Depression" was published in 2022. Journal: Evid Based Complement Alternat Med.

#### 2.5.4. Female Urine Sniffing Test (FUST)

The mice were habituated to a sterile cotton-tipped applicator that was placed into their home cage for 1 hour. Then, each mouse was exposed to two cotton-tipped applicators, one dipped in water and the other dipped in the urine of female estrus, in a quiet, dimly lit room (<20 lux). This test lasted for 3 minutes, and the time the mice spent sniffing each cotton tip was measured.

#### 2.5.5. Elevated Plus Maze (EPM)

This apparatus consisted of a cross-shaped maze with two oppositely positioned arms, one open and one closed, with a 5 cm × 5 cm center. The device was a white opaque Plexiglas maze 40 cm above the ground; each arm was 30 cm × 5 cm × 30 cm. The mice were placed in the center of the maze with their heads facing the open arm. Their movement was filmed for 5 minutes, and the time they spent in the open arm was measured using video-tracking software (Smart 3.0, Panlab, Spain).

#### 2.5.6. Open Field Test (OFT)

The OFT was conducted in dimly illuminated conditions in a white opaque Plexiglas chamber (50 × 50 × 40 cm). The mice were gently placed inside the chamber, and their movements were filmed for an hour and analyzed using video-tracking software (Smart 3.0, Panlab, Spain). The chamber device inside was cleaned with 70% ethanol after each experiment.

#### 2.5.7. Sucrose Preference Test (SPT)

The SPT was based on the sucrose preference ratio of rodents, with reference to the study by Liu et al. [40]. Mice were exposed to two identical bottles overnight from 19:00 to 10:00 the next morning: one bottle contained water and the other contained a 1% sucrose solution. Both bottles were weighed before and after this period, and the sucrose preference was calculated as the ratio of the volume of sucrose to the total volume of sucrose and water consumed.

### 2.6. Western Blotting

Animals were deeply anesthetized and then rapidly sacrificed. Their dissected prefrontal cortex and hippocampus tissues were stored at −80°C until use. Tissues were homogenized with lysis buffer containing 1% each of phosphatase inhibitor cocktails 2 and 3 (P5726, P044, Sigma-Aldrich) in PRO-PREP™ (17081, iNtRON Biotechnology, Seongnam, South Korea) and centrifuged at 13,000 rpm for 10 minutes at 4°C. Protein concentrations were measured using DC™ Protein Assay Reagents A, B, and S (5000113, 5000114, and 5000115, BIO-RAD, Hercules, CA, USA). After electrophoresis using 10% SDS-polyacrylamide gel, the gel phase proteins were transferred to a nitrocellulose membrane (162-0115, BIO-RAD). Membranes were incubated for 1 hour at room temperature in 5% nonfat dry milk (170-6404, BIO-RAD) dissolved in TBS-T (0.1% tween 20 in TBS) for blocking. Primary antibodies were diluted in 5% nonfat dry milk in TBS-T and incubated overnight at 4°C. The next day, the membranes were washed thrice for 10 minutes with TBS-T. Secondary antibodies were diluted with 5% nonfat dry milk in TBS-T and incubated for 1 hour at room temperature. After washing thrice for 10 minutes with TBS-T, luminescence was induced using a Pierce™ ECL Western Blotting Substrate Kit (32106, Thermo Fisher Scientific, Waltham, MA, USA), and the samples were photographed with an EZ-Capture MG (ATTO, Tokyo, Japan). Band density was analyzed using ImageJ software (NIH, Bethesda, MD, USA). The antibodies used in this experiment were mTOR (#2972, 1:1000, Cell Signaling), p-mTOR (Ser2448, #2971, 1:1000, Cell Signaling), GluR1 (AP08676, 1:2500, Tocris), p-GluR1 (Ser845, #8084, 1:1000, Cell Signaling), beta-actin (sc-47778, 1:5000, Santa Cruz), anti-rabbit IgG (H + L) HRP conjugate (W4011, 1:1000, Promega, Madison, WI, USA), and anti-mouse IgG (H + L) HRP conjugate (W4021, 1:5000, Promega).

The article "Rapid-Onset Antidepressant-Like Effect of Nelumbinis semen in Social Hierarchy Stress Model of Depression" was published in 2022. Journal: Evid Based Complement Alternat Med.

### 2.7. Statistical Analysis

The results are expressed as the mean ± SEM. Statistical comparisons were performed using unpaired T-testing (SPT) or one-way ANOVA (TST, FST, OFT, EPM, FUST, and NSFT) followed by LSD or Tukey's HSD post hoc multiple comparisons testing using SPSS 22 (SPSS Inc., Chicago, IL, USA). A *p* value <0.05 was considered statistically significant.

## 3. Results

### 3.1. Antidepressant-Like Effect of NS in Normal Mice (Cohort 1)

Behavioral measurements were performed in normal mice to test the antidepressant effect of NS (cohort 1). After acclimatizing to the environment for 7 days, each mouse was given one of three different doses of NS (0.1 mg/kg, 1 mg/kg, or 10 mg/kg), and the effects were measured using the NSFT, TST, FST, FUST, EPM, and OFT, as described in the methods and depicted in Figure 1.

In the NSFT, there were no differences among the experimental groups in the latency to feed (Figure 2(a)). In the TST, immobility was reduced by NS 0.1 mg/kg and 1 mg/kg compared with the control (Figure 2(b)), but the immobility reduction in the NS 10 mg/kg group was insignificant (*p*=0.228). In the FST, immobility was reduced in all the NS-treated groups (Figure 2(c)). Among the NS doses, 1 mg/kg was the most effective. In the FUST, EPM, and OFT, no NS dose changed the behavioral responses (Figures 2(d)∼2(f)) except that the 10 mg/kg group had higher locomotor activity than the 0.1 mg/kg group in the OFT (*p*=0.007). These results indicate that NS might have antidepressant-like (but not anxiolytic) and activity-stimulating effects. Presenting better performance, 1 mg/kg of NS was used for further experiments.

The article "Rapid-Onset Antidepressant-Like Effect of Nelumbinis semen in Social Hierarchy Stress Model of Depression" was published in 2022. Journal: Evid Based Complement Alternat Med.

### 3.2. Antidepressant Effect of NS in the Social Hierarchy Stress Model (Cohort 2)

Behavioral measurements were made for SHS depression model mice to test the antidepressant effect of NS (cohort 2). SHS was performed as described in the methods, and the effects of NS 1 mg/kg were compared with the effects of fluoxetine 10 mg/kg using the SPT, NSFT, TST, FST, FUST, EPM, and OFT, as depicted in Figure 1.

In the SPT, the sucrose preference in the SHS-exposed animals decreased, indicating that the SHS established a depression-like state in those mice (Figure 3(a)). In further experiments, DW (in the normal and vehicle groups) and NS 1 mg/kg were administered orally, and fluoxetine 10 mg/kg was injected intraperitoneally 30 minutes before each test. In the TST, immobility increased following SHS (normal vs. vehicle-treated SHS), and NS but not fluoxetine reduced the immobility of mice exposed to SHS (Figure 3(b)). In the FST, immobility also increased following SHS (normal vs. vehicle-treated SHS), and NS but not fluoxetine reduced that immobility (Figure 3(c)). In the FUST, the time spent smelling distilled water did not differ between the groups, but NS increased the time the SHS-exposed mice spent smelling estrus female urine (Figure 3(d)).

In the EPM, the anxiety-related behaviors did not change (Figure 4(a)). Likewise in the OFT, the locomotor activity did not differ among the experimental groups (Figure 4(b)). But in the NSFT, the latency to eat a pellet, which is an anxiety-related response, was prolonged in the SHS-exposed mice and reduced by NS (Figure 4(c)). No anxiety-related changes were detected in the EPM, which suggests an antidepressant effect.

### 3.3. AMPA Receptor Dependency of the Antidepressant-Like Effects of NS (Cohort 3)

Behavioral measurements were performed in normal mice to evaluate the antidepressant effects of NS in relation to the AMPA receptor (cohort 3). After acclimatizing to the environment for 7 days, each mouse was given NS 1 mg/kg with or without NBQX (AMPA antagonist), and the effects were measured using the NSFT, TST, FST, and FUST, as depicted in Figure 1.

In the NSFT, feeding latency was shortened by NS. Although NBQX did not affect the feeding latency in untreated mice, it blocked the latency shortening effect of NS (Figure 5(a)). In the TST and FST, NBQX blocked the immobility-reducing effects of NS (Figures 5(b) and 5(c)). Also, NBQX blocked the NS-induced increase in the hedonic-like response to female urine (Figure 5(d)).

The article "Rapid-Onset Antidepressant-Like Effect of Nelumbinis semen in Social Hierarchy Stress Model of Depression" was published in 2022. Journal: Evid Based Complement Alternat Med.

### 3.4. Involvement of mTOR and GluR1 Signaling in the Antidepressant-Like Effect of NS

Because NS demonstrated the possibility of acute-onset antidepressant-like properties, mTOR and GluR1, which are molecular signals related to acute-onset antidepressant effects, were measured in the prefrontal cortex and hippocampus tissues extracted from the cohort 3 mice.

In the prefrontal cortex, phospho-mTOR was increased by NS, and that increase was blocked by NBQX cotreatment (Figures 6(a) and 6(b)). However, the differences in total mTOR expression among groups were nonsignificant. In the hippocampus, no changes were detectable in the total or phospho forms of mTOR expression (Figures 6(d) and 6(e)).

In the prefrontal cortex, the total and phosphor-GluR1 expression was unaltered (Figures 7(a) and 7(b)). In the hippocampus, the total expression of GluR1 was not altered by NS or NBQX (Figure 7(d)), but the amount of phosphor-GluR1 in the hippocampus decreased after NS treatment (Figure 7(e)).

## 4. Discussion

To examine the antidepressant-like and rapid-onset antidepressant-like actions of NS, we conducted behavioral tests and biochemical analyses in normal and depression-model mice. We found that NS reduced the behavioral despair of normal mice in the range of 0.1 to 10 mg/kg, reduced behavioral despair and increased hedonic behavior in SHS-exposed mice, and showed rapid-onset antidepressant-like effects in the NSFT. Blockade of the AMPA receptor inhibited the antidepressant-like activity of NS. Also, NS increased the phosphorylation of mTOR in the prefrontal lobe and reduced the phosphorylation of GluR1-845 in the hippocampus.

NS has been widely used in oriental traditional medicine as a remedy for insomnia, anxiety, and depression [14]. Many preclinical studies have demonstrated its antidepressant-like effects since the discovery of serotonergic receptor ligands in this herbal medicine [41]. In nonstressed rats, three intraperitoneal injections of NS given at 400 mg/kg exerted antidepressant-like effects in the FST, but the effects of other doses (100, 200, and 1000 mg/kg) were insignificant [14]. Another study demonstrated that among the different solvents used to prepare NS extracts, the n-butyl alcohol extract showed the strongest inhibitory effect on immobility in the FST in normal rats [42]. It was suggested that NS might exert an antidepressant effect by enhancing serotonin [43].

Unlike previous studies, we tested the antidepressant effect of NS in a dose range of 0.1 to 10 mg/kg because the dose of ketamine that produces rapid-onset antidepressant effects is 10 mg/kg, which is much lower than the dose that causes anesthetic effects. Similarly, *Radix polygalae*, which also produces rapid-onset antidepressant-like effects, is effective at a dose of 1 mg/kg [7,44]. We found that NS reduced despair behaviors in the TST and FST after a single administration of 0.1 mg/kg and 1 mg/kg, and it reduced despair behavior in the FST at 10 mg/kg. In that dose range, NS had no anxiolytic- or psychomotor-stimulating effects. Also, it had no effect on the pleasure-seeking behavior evaluated in the FUST. Decreased pleasure-seeking behavior is one of the main symptoms of depression, and due to ceiling effects, NS might not have increased pleasure-seeking behavior in nondepressed animals. According to previous studies, NS had an antidepressant-like effect at a high dose (400 mg/kg) that is related to serotonergic signaling. Our results suggest an antidepressant-like effect at a low dose (0.1 to 10 mg/kg) showing a possibility that the antidepressant-like effects of NS are biphasic.

The article "Rapid-Onset Antidepressant-Like Effect of Nelumbinis semen in Social Hierarchy Stress Model of Depression" was published in 2022. Journal: Evid Based Complement Alternat Med.

Several methods are used to create models of depression in animals, but most commonly, stressors are applied to induce depression-like behaviors. Such methods have high construct validity in that long-term stress induces depression. However, animal models often use physical stressors, whereas the stress that people endure is often psychosocial. Therefore, depression models that use social stressors may be more valid and could reduce the gap between animal and clinical studies. As a model of social stress, the social defeat model is widely used, but we used the social hierarchy model because the social defeat model exposes animals to direct violence during the resident-intruder paradigm, which means that physical stress has a great influence on the formation of the model. In the SHS model, on the other hand, the depressed state is induced through frustration rather than exposure to direct physical harm. This method models experiences such as being pushed out of being an alpha male in chimpanzee society and celebrities moving away from public attention in human life, which is more appropriate than a social defeat for a depression model because depression occurs more often in those conditions rather than by becoming a victim of violence.

In mice exposed to SHS stress, anhedonia, measured as the preference for sweet water and time spent sniffing the urine of an estrus female, and despair behavior, measured using the FST and TST, were increased. Also, the latency to feeding was increased in the NSFT, but anxiety-like behavior and general activity did not change. Latency in the NSFT measures anxiety-like and depression-like behaviors, and locomotor activity can affect its outcome [32,45]. Because the anxiety and locomotor activity levels did not change, SHS induced a depressive phenotype in the mice.

The article "Rapid-Onset Antidepressant-Like Effect of Nelumbinis semen in Social Hierarchy Stress Model of Depression" was published in 2022. Journal: Evid Based Complement Alternat Med.

When the effects of NS and fluoxetine were tested in this animal model of depression, a single dose of NS, but not a single dose of fluoxetine, reduced despair and anhedonic behaviors. Neither NS nor fluoxetine had any effect on anxiety or locomotion, but NS (but not fluoxetine) reduced the latency to feeding in the NSFT. This is also an antidepressant-like effect because NS did not affect anxiety or locomotion. In previous studies, the anti-anxiety effect of NS was detected in animals treated with normal and chronic unpredictable mild stress [25,46]. However, the doses of NS in those studies were 50 to 400 mg/kg, much higher than those we used in this study. Therefore, because low-dose NS did not affect anxiety or locomotion, the shortening of latency in the NSFT was an antidepressant-like effect. On the other hand, fluoxetine did not show any such antidepressant-like effect, and it is known that in the NSFT, fluoxetine exhibits antidepressant effects only when it is administered chronically [32,45,47]. Therefore, SHS seems to be a model for depression that responds to chronic administration of antidepressants, and NS seemed to exhibit rapid-onset antidepressant action in that model. So, our next step was to test its rapid-onset antidepressant effect.

To verify the rapid-onset antidepressant-like effect of NS, we pretreated mice with NBQX to block the AMPA receptor before behavior tests. An AMPA receptor blockade is known to abolish the rapid-onset antidepressant action of drugs that act on the glutamatergic system [8] such as ketamine, rapastinel, LY314597, (2R,6 R)-HNK, and scopolamine [48]. In our results, administration of NBQX alone did not affect depressive behaviors, but it suppressed the antidepressant effect of NS. In the NSFT, the reduced feeding latency seen with NS was blocked by NBQX pretreatment. As shown in Figure 4, the reduced latency in the NSFT caused by NS was not related to anxiety or spontaneous locomotion; therefore, NBQX blocked the rapid-onset antidepressant-like effect of NS. The despair response reduction caused by NS in the FST and TST was also blocked by NBQX. This result is parallel to that seen with ketamine [8,49]. In addition, the increase in urine sniffing time in the FUST was blocked by NBQX, indicating that the AMPA receptor blockade inhibited the hedonic-like behavior induced by NS.

A rapid-onset antidepressant effect is generally known to have a relationship with mTOR signaling, so mTOR phosphorylation was measured in the prefrontal cortex and hippocampus after NS administration. As expected, phosphorylated mTOR was increased by NS, and that effect was blocked by NBQX in the prefrontal cortex. The difference in the total amount of mTOR expressed in the prefrontal cortex was not statistically significant, and there was no difference in the amount of phosphorylated and total mTOR expressed in the hippocampus.

The article "Rapid-Onset Antidepressant-Like Effect of Nelumbinis semen in Social Hierarchy Stress Model of Depression" was published in 2022. Journal: Evid Based Complement Alternat Med.

Li et al. found that the rapid antidepressant action of ketamine was due to an increase in phosphorylated mTOR in the prefrontal cortex [7], which indicates the synapse enhancement through mTORC1 signaling that has also been correlated with the rapid-onset antidepressant effect of Ro 25-6981 [7], mGluR2/3 antagonists [50], (2R,6R)-hydroxynorketamine [51], rapastinel [52], and scopolamine [53]. Such antidepressant effects also appear upon the activation of the p70S6 kinase, a downstream effector of mTORC1, or sestrin [48,54]. Studies have reported that mTOR phosphorylation is increased in the ventral hippocampus but not in the dorsal hippocampus [55]. In a schizophrenia model, the administration of 60 mg/kg of ketamine twice a day for 7 days decreased mTOR expression in the prefrontal cortex and hippocampus [56]. In our experimental results, the antidepressant action of NS appears to be related to mTOR phosphorylation in the prefrontal cortex but not in the hippocampus. However, it could be that no difference was found in the hippocampus because of measuring in the entire hippocampus instead of dividing it into ventral and dorsal parts.

It is known that rapid antidepressant action is associated with changes in AMPA receptors. Ketamine rapidly increases GluR1 expression in synaptosomes of the prefrontal cortex [7]. Antidepressant effect of ketamine was blocked by an AMPA receptor blockade, and phosphorylation of the GluR1 subunit was reduced [8]. In our results, the expression level and phosphorylated form of GluR1 were not affected by NS in the prefrontal cortex, but the phosphorylated form of GluR1 was reduced in the hippocampus. Ketamine was reported to reduce p845 on the GluR1 receptor subunit in the hippocampus [57], and similarly, an mGluR7 agonist with rapid-onset antidepressant action also reduced the p845 of GluR1 [58].

Phosphorylation of S845 and S831 on the GluR1 subunit regulates the membrane expression of AMPA receptors [59]. In stress-induced depression models, the phosphorylation of S845 was decreased in some articles and increased in others [60,61]. When antidepressants such as imipramine and tianeptine were administered, the phosphorylation of S845 in the hippocampus increased [62,63]. Therefore, more research is needed to determine whether the results of this study fit the pharmacological mechanism of antidepressants in terms of the phosphorylation of GluR1 subunits. Also, the antidepressant effect of NS was found to have different actions in the prefrontal cortex and hippocampus.

The article "Rapid-Onset Antidepressant-Like Effect of Nelumbinis semen in Social Hierarchy Stress Model of Depression" was published in 2022. Journal: Evid Based Complement Alternat Med.

One concern in this study was that the number of animals in the SHS model group was only 4, which was smaller than that of general animal behavioral experiments. This is because four times as many animals are needed to make SHS depression model mice. However, the mice induced with SHS showed a clear difference compared with the normal mice in sucrose preference, and the SHS mice treated with NS and fluoxetine also showed a clear difference from the untreated SHS mice. This effect was verified statistically as the *p* value below 0.05 indicates a good chance of difference in the distribution of data values.

## 5. Conclusions

NS reduced behavioral despair in the FST and TST. Under the condition of SHS, hedonic behavior was reduced, the despair response was increased, and the time to approach food in the NSFT was longer, indicating a condition of depression. Under the SHS condition, NS but not fluoxetine reduced those depression-like behaviors. Specifically, NS showed a rapid antidepressant-like effect by acutely reducing the access time to the food pellet in the NSFT. The administration of NBQX, an AMPA receptor blocker, inhibited the antidepressant-like effect of NS in the FST, TST, and NSFT, and the effects of NS were related to enhanced phosphorylation of mTOR in the prefrontal cortex and dephosphorylation of GluR1 S845 in the hippocampus. When the NS dose was increased, the tendency of the antidepressant effects to decrease was similar to that found with ketamine. Since NS has shown antidepressant-like potential in a preclinical model, it may be considered as a research candidate for the development of antidepressants in the future.

## Figures and Tables

**Figure 1:** Schematic diagram of the experimental outline. NS (*Nelumbinis semen*), NSFT (novelty suppressed feeding test), TST (tail suspension test), FST (forced swim test), FUST (female urine sniffing test), EPM (elevated plus maze), OFT (open field test), SPT (sucrose preference test), and DW (distilled water).

**Figure 2:** Antidepressant-like effects of *Nelumbinis semen* (NS). Tests were performed 30 minutes after NS administration (0.1, 1, and 10 mg/kg p.o.). (a) Novelty suppressed feeding test: the latency to feed did not differ among the groups (*F*(3,20) = 1.718, *p*=0.195). (b) Tail suspension test: immobility time changed significantly (*F*(3,20) = 3.685, *p*=0.029). Immobility was reduced in the 0.1 mg/kg (*p*=0.038) and 1 mg/kg (*p*=0.047) groups relative to the vehicle group. (c) Forced swim test: immobility time changed significantly (*F*(3,20) = 7.229, *p*=0.002). Immobility was reduced in the 0.1 mg/kg (*p*=0.036), 1 mg/kg (*p*=0.004), and 10 mg/kg (*p*=0.039) groups relative to the vehicle group. (d) Female urine sniffing test: the time spent sniffing DW (*F*(3,20) = 1.988, *p*=0.148) and estrus female urine (*F*=(3,20) = 2.042, *p*=0.140) did not differ among the experimental groups. (e) Elevated plus maze: time spent in the open arm was not significantly changed (*F*(3,20) = 0.688, *p*=0.57). (f) Open field test: distance moved in the open field differed among the groups (*F*(3,20) = 4.976, *p*=0.01), but there were no significant changes compared with the vehicle group. Data are shown as the mean ± SEM (*n* = 6/group). Vehicle: distilled water p.o.; 0.1 mg/kg: NS 0.1 mg/kg p.o.; 1 mg/kg: NS 1 mg/kg p.o.; and 10 mg/kg: NS 10 mg/kg p.o.; ^*∗*^*p* < 0.05, ^*∗∗*^*p* < 0.01 vs. vehicle. ANOVA, Tukey's HSD post hoc test.

The article "Rapid-Onset Antidepressant-Like Effect of Nelumbinis semen in Social Hierarchy Stress Model of Depression" was published in 2022. Journal: Evid Based Complement Alternat Med.

**Figure 3:** Antidepressant-like effect of *N. semen* (NS) measured in social hierarchy stress (SHS) depression model mice. Tests were performed 30 minutes after NS (1 mg/kg p.o.) or fluoxetine (10 mg/kg i.p.) administration. (a) Sucrose preference test: sucrose preference (%) was reduced in SHS-exposed mice compared with unexposed normal mice (*p*=0.001). (b) Tail suspension test: immobility time differed significantly among groups (*F*(3,12) = 17.264, *p* < 0.001). The immobility time in the SHS animals increased (normal vs. vehicle, *p*=0.013). NS reduced the immobility in the SHS model animals (vehicle vs. NS, *p* < 0.001), but fluoxetine did not (vehicle vs. fluoxetine, *p*=0.507). (c) Forced swim test: immobility time differed significantly among groups (*F*(3,12) = 26.584, *p* < 0.001). Following SHS exposure, immobility increased compared with normal mice (normal vs. vehicle, *p* < 0.001). NS reduced the immobility in SHS model animals (vehicle vs. NS, *p*=0.004), but fluoxetine did not (vehicle vs. fluoxetine, *p*=0.926). (d) Female urine sniffing test: the time spent sniffing distilled water did not differ among the groups (*F*(3,12) = 1.53, *p*=0.257), but the time spent sniffing the urine differed significantly (*F*(3,12) = 3.534, *p*=0.048). The vehicle group spent less time sniffing the urine, but the difference was not significant (normal vs. vehicle, *p*=0.143). Sniffing time was increased by NS in the SHS-exposed mice (*p*=0.041). Data are shown as the mean ± SEM (*n* = 4). Normal: not exposed to SHS; SHS: exposed to social hierarchy stress; vehicle: SHS + distilled water p.o.; NS: SHS + NS 1 mg/kg p.o.; fluoxetine: SHS + fluoxetine 10 mg/kg i.p.; ^*∗*^*p* < 0.05, ^*∗∗*^*p* < 0.01, ^*∗∗∗*^*p* < 0.001 vs. normal; ^#^*p*<0.05, ^###^*p*<0.001 vs. vehicle. Student's t-test for (a), and ANOVA and Tukey's HSD post hoc test for (b), (c), and (d).

The article "Rapid-Onset Antidepressant-Like Effect of Nelumbinis semen in Social Hierarchy Stress Model of Depression" was published in 2022. Journal: Evid Based Complement Alternat Med.

**Figure 4:** Acute-onset antidepressant-like effects of *Nelumbinis semen* (NS) measured using the social hierarchy stress (SHS) depression model. Tests were performed 30 minutes after NS (1 mg/kg p.o.) or fluoxetine (10 mg/kg i.p.) administration. (a) Elevated plus maze: the time spent in the open arm did not differ significantly among the experimental groups (*F*(3,12) = 0.598, *p*=0.625). The reduced open-arm time in the fluoxetine group was insignificant (vehicle vs. fluoxetine, *p*=0.675). (b) Open field test: the travel distance did not differ among the groups (*F*(3,12) = 0.262, *p*=0.852). (c) Novelty suppressed feeding test (NSFT): the latency to take a food pellet differed significantly among the groups (*F*(3,12) = 4.999, *p*=0.018). The latency increased in the SHS animals (normal vs. vehicle, *p*=0.046). NS reduced the latency in the SHS animals (vehicle vs. NS, *p*=0.019), but fluoxetine did not (vehicle vs. fluoxetine, *p*=0.081). Data are shown as the mean ± SEM (*n* = 4). ^*∗*^*p* < 0.05 vs. normal, ^#^*p* < 0.05 vs. vehicle. ANOVA, Tukey's HSD post hoc test.

**Figure 5:** The role of the *α*-amino-3-hydroxy-5-methylisoxazole-4-propionic acid (AMPA) receptor in the antidepressant-like effect of *N. semen* (NS). Behavioral tests were performed 40 minutes after NBQX injection (10 mg/kg, i.p.) and 30 minutes after NS administration (1 mg/kg p.o.). (a) Novelty suppressed feeding test: there was no interaction between NS and NBQX (*F*(1,20) = 3.882, *p*=0.063), but there was a main effect of NS (*F*(1,20) = 8.613, *p*=0.008) and NBQX (*F*(1,20) = 11.201, *p*=0.003). Latency to take a food pellet was reduced by NS (*p*=0.012), and that reduction was blocked by NBQX (*p*=0.006). (b) Tail suspension test: there was a group difference (*F*(3,20) = 5.894, *p* < 0.005) and an NS^*∗*^NBQX interaction (*F*(1,20) = 13.828, *p*=0.001). Immobility time was reduced in the NS group (*p*=0.007 vs. vehicle), and the reduction in immobility caused by NS was blocked by NBQX (*p*=0.011). (c) Forced swim test: NBQX had a significant main effect (*F*(1,20) = 13.503, *p*=0.002) and NS^*∗*^NBQX interaction (*F*(1,20) = 30.266, *p* < 0.001). The immobility was reduced by NS (*p* < 0.001), and that effect was blocked by NBQX (*p* < 0.001). (d) Female urine sniffing test: the time spent sniffing distilled water did not differ between the groups, but the time spent sniffing estrus female urine increased significantly in the NS group relative to the vehicle group (*p*=0.012), and that antidepressant-like effect was reduced by NBQX (*p*=0.001). There was also an NS^*∗*^NBQX interaction in the time spent sniffing urine (*F*(1,20) = 13.828, *p*=0.001). Data are shown as the mean ± SEM (*n* = 6). ^*∗*^*p* < 0.05, ^*∗∗*^*p* < 0.01, ^*∗∗∗*^*p* < 0.001 vs. vehicle, ^#^*p*<0.05, ^##^*p*<0.01, ^###^*p*<0.001 vs. NS. Two-way ANOVA, Tukey's HSD post hoc test.

The article "Rapid-Onset Antidepressant-Like Effect of Nelumbinis semen in Social Hierarchy Stress Model of Depression" was published in 2022. Journal: Evid Based Complement Alternat Med.

**Figure 6:** Effects of *Nelumbinis semen* (NS) and AMPA blockade on mTOR expression in the prefrontal cortex (PFC) and hippocampus. (a) Normalized mTOR/*β*-actin of PFC:  there was a significant change among groups (*F*(3,20) = 4.723, *p*=0.012), but mTOR levels were nonsignificantly increased by NS (*p*=0.064), and NBQX did not affect the expression of mTOR in the NS-treated animals (*p* = 0.095*p*=0.095). (b) Normalized phospho-mTOR/*ß*-actin of PFC: there was a significant change among groups (*F*(3,20) = 2.613, *p*=0.008). p-mTOR expression increased with NS treatment compared with vehicle (*p*=0.026), and NBQX decreased the p-mTOR expression in NS-treated animals (*p*=0.03). (c) Representative blot image of total and phospho-mTOR expression in the PFC. (d) Normalized mTOR/*ß*-actin of the hippocampus: there was no significant change among groups (*F*(3,20) = 0.428, *p*=0.735). (e) Normalized phospho-mTOR/*ß*-actin of the hippocampus. There was no significant change among groups (*F*(3,20) = 0.383, *p*=0.767). (f) Representative blot image of total and phosphor-mTOR expression in the hippocampus. The parentheses in (c) and (f) correspond to the treatments indicated above them. Data are shown as the mean ± SEM (*n* = 6). ^*∗*^*p* < 0.05 vs. vehicle, ^#^*p* < 0.05 vs. NS. ANOVA, LSD post hoc test.

**Figure 7:** Effects of *Nelumbinis semen* (NS) and AMPA blockade on GluR1 expression in the prefrontal cortex (PFC) and hippocampus. (a) Normalized GluR1/*ß*-actin of PFC: there was no significant change (*F*(3,20) = 1.145, *p*=0.259). (b) Normalized phospho-GluR1/*ß*-actin of PFC: there was no significant change (*F*(3,20) = 0.517, *p*=0.675). (c) Representative blot image of the total and phospho-GluR1 expression in the PFC. The parentheses correspond to the treatments indicated above them. (d) Normalized GluR1/*ß*-actin of the hippocampus: ANOVA revealed no significant differences among groups (*F*(3,20) = 2.692, *p*=0.074). (e) Normalized phospho-GluR1/*ß*-actin of the hippocampus: the phospho-GluR1 levels changed significantly (*F*(3,20) = 4.48, *p*=0.024). Phospho-GluR1 decreased with NS treatment (*p*=0.04), but the difference between the NS and NS + NBQX groups was nonsignificant. (f) Representative blot image of the total and phospho-GluR1 expression in the hippocampus. The parentheses in (c) and (f) correspond to the treatments indicated above them. Data are shown as the mean ± SEM (*n* = 6). ^*∗*^*p* < 0.05 vs. vehicle, ^#^*p* < 0.05 vs. NS. Non-sig: nonsignificant. ANOVA, LSD post hoc test.

The article "Rapid-Onset Antidepressant-Like Effect of Nelumbinis semen in Social Hierarchy Stress Model of Depression" was published in 2022. Journal: Evid Based Complement Alternat Med.

## Data Availability

The data used to support the findings of this study are available from Seung-Yun Cha upon your request.
